The article "Astragaloside IV ameliorates fat metabolism in the liver of ageing mice through targeting mitochondrial activity" was retracted in 2025. Reasons: plagiarized images; duplicated images; overlap with other authors' work; unreliable results or conclusions.

# Astragaloside IV ameliorates fat metabolism in the liver of ageing mice through targeting mitochondrial activity

**DOI:** 10.1111/jcmm.16847

**Published:** 2021-08-17

**Authors:** Zhixiao Luo, Yaqi Wang, Mengzhen Xue, Fangqi Xia, Leiqi Zhu, Yuanyang Li, Dengke Jia, Silong Chen, Guangfu Xu, Yan Lei

**Affiliations:** ^1^ Health Management Center The First Affiliated Hospital of Chongqing Medical University Chongqing China; ^2^ College of Medical Science China Three Gorges University Yichang China; ^3^ Department of Otorhinolaryngology The First Affiliated Hospital of Chongqing Medical University Chongqing China

**Keywords:** ageing, Astragaloside IV, energy metabolism, fat catabolism, mitochondria, respiratory quotient, β‐oxidation

## Abstract

Astragaloside IV (AST) is a major bioactive compound of *Radix Astragali* with medical and health benefits. Previous studies have found that AST can reduce the body weights of high‐fat diet fed mice. However, the effect of AST on fat metabolism of ageing mice is unclear. In this study, naturally ageing mice were administered intragastrically with AST at 30 mg/kg/day (ageing + AST‐L group) and 90 mg/kg/day (ageing + AST‐H group) for 16–20 months. Adult (4 months old) and ageing mice were given 1% sodium carboxyl methylcellulose as vehicle. Energy metabolism‐related biological parameters of living mice were examined. Moreover, mRNA and protein levels of key enzymes/proteins involved in triglyceride (TG) lipolysis, fatty acid β‐oxidation (FAO), ketone body (KB) production and mitochondrial respiratory chain were also examined after sacrifice. Results demonstrated that treatment with AST significantly reduced body weight, white fat and liver/body weight ratio of ageing mice, significantly reduced serum/hepatic TG levels, respiratory quotient, promoted fatty acid mobilization in white adipose tissue, mitochondrial FAO and KB production and mitochondrial biosynthesis/functions in the liver of ageing mice. AST also up‐regulated the expression of phosphorylated AMP‐activated protein kinase, acetyl‐CoA carboxylase, acetyl‐coenzyme A synthetase, carnitine palmitoyltransferase 1a/1b, enoyl coenzyme A hydratase‐short chain, acyl‐CoA dehydrogenase medium chain and mitochondrial 3‐hydroxy‐3‐methylglutaryl‐CoA synthase‐2 involved in fat metabolism. These results indicated that mitochondrial activity could be the target of AST to treat abnormal fat metabolism during ageing.

## 1 INTRODUCTION

Ageing is a time‐dependent process and controlled by multiple factors, involving the changes in different physiological systems and the complex interactions among genetic, epigenetic, environmental factors and the alterations in the gut microbiome.^1^, ^2^ With the body ageing, the physiological functions of most organs are decreased, and the morbidity rate and mortality rate are increased due to different diseases. The susceptibility of the aged to pathogenic infections is also increased.^3^ With the increase of human life span, the ageing‐related morbidity and the declined organ functions have become a serious public health problem globally. Whether there are safer and more sufficient medical and economic resources to effectively deal with the increasing elderly population suffering from a variety of ageing‐related diseases and the declined immunity is becoming a serious socio‐economic problem.^4^ Achieving a better and healthier living in old age is one of the biggest challenges in our current society. To promote more studies on ageing and ageing‐related diseases and to develop functional foods for treatment of ageing‐related diseases can be the practical way to improve healthy and productive longevity for the elderly population.^4^ The prevalence of senile obesity caused by the declined body's metabolic functions associated with ageing is increasing. In the process of ageing, the body's basal metabolic rate decreases, and fat content is increased, accumulated and distributed abnormally, resulting in the increased visceral adipose tissue (VAT), accompanied by dyslipidaemia and other obesity symptoms. However, currently, the effective clinical treatments for this clinical problem have not been available. Recent studies have shown that traditional Chinese medicines (TCMs) are quite effective in delaying ageing and improving ageing‐related abnormalities of lipid metabolism. A number of phytochemicals have been known to be beneficial on age‐related diseases.^5^ For instance, resveratrol, a type of phenol and a phytoalexin naturally produced by plants, can improve the abnormalities of lipid metabolism caused by ageing and reduce ageing‐caused weight gain and the increased level of blood TG.^6^ Quercetin, an antioxidant found in apples and other types of foods, is also effective on delaying metabolic abnormalities caused by ageing.^7^ Therefore, to conduct an in‐depth study on the TCM‐intervention and its mechanism of abnormal lipid metabolism caused by ageing is of great significance for the prevention and treatment of senile obesity.^8^, ^9^, ^10^

The liver is the central organ for TG and fatty acid metabolism. Abnormal lipid metabolism is closely related to the abnormal liver functions. The main feature of a common disease in the liver, such as non‐alcoholic fatty liver disease (NAFLD), is resulted from the abnormal TG accumulation in the liver. Increasing lines of evidence have indicated that ageing is an important risk factor for the development of NAFLD.^11^, ^12^, ^13^ The TG accumulation in the liver of senile patients is mainly caused by the imbalance of their synthesis and clearance. The catabolism of free fatty acids (FFAs) in hepatocytes is mainly regulated by the mitochondrial FAO system. The abnormal mitochondrial FAO in liver cells is generally considered to be the main mechanism of abnormal lipid metabolism in the liver and even the entire body. Clinical studies have also shown that patients with abnormal lipid metabolism in the body usually have mitochondrial dysfunction and FAO damage in their liver.^14^ Therefore, to improve mitochondrial functions and mitochondrial FAO has become a potential new direction for developing the treatment measures for the abnormal lipid metabolism in the ageing body.

Astragali radix is one of the most commonly used TCMs. It is generally extracted from the dried root of *Astragalus mongholicus Bunge* (*A*. *mongholicus*). In Europe, the Middle East and Asia, it is widely used in coffee, food and tea substitutes.^15^, ^16^ Currently, astragalus‐derived products, such as astragalus tea and food additives, can be sold in the US health food market.^17^ Astragalus‐jujube‐wolfberry tea is a well‐known tea in China, which possesses anti‐cancer activity, can improve immunity and enhance body viability.^18^ In addition, Astragali radix confers a variety of stimulatory effects, including immune regulation, antioxidation, anti‐tumour, anti‐viral, diuretic, lowering blood sugar and lowering blood lipids.^19^, ^20^ Recent studies have shown that Astragali radix has therapeutic effects on neurodegenerative diseases as well.^21^ Particularly, Astragaloside IV (AST) is a natural saponin molecule and one of the main active components of Astragalus. AST has been reported to have a variety of pharmacological activities, including antioxidation, anti‐inflammation, anti‐diabetes and hypertension activities.^22^, ^23^, ^24^, ^25^, ^26^ However, little is known regarding whether AST can affect mitochondrial FAO and energy metabolism in the liver of ageing mice. Therefore, in the present study, we aimed to test our hypothesis that AST is capable of effectively regulating mitochondrial FAO and energy metabolism in healthy ageing mice by mainly regulating the activation of fatty acids in the liver and transport into mitochondria, enhancing mitochondrial FAO and mitochondrial biosynthesis and functions of liver of ageing mice.

## 2 MATERIALS AND METHODS

### 2.1 Mice and AST administration

Forty naturally ageing C57BL/6J male mice were purchased from Beijing Vital River Laboratory Animal Technology Co., Ltd with animal certificate number No. SCXK (Beijing) 2016‐0006. The mice were maintained in separate cages in the Experimental Animal Center of China Three Gorges University (Yichang, Hubei, China), at room temperature (22 ± 2)°C, humidity (60 ± 5) %, alternating light and dark for 12 h, with free access to water drinking and food eating. All the mouse experiments were performed in compliance with the Laboratory Animal Operating Standards of China Three Gorges University, and the animal protocols were approved by the Institute's Ethics Committee (Nọ: 2017030E). The mice were randomly divided into four groups: 4 months old (adult group), 20 months old (ageing group), 20 months old with treatment of Astragaloside IV (AST) at low‐dose group (AST‐L group), and 20 months old with AST treatment at high‐dose group (AST‐H group) with 10 mice in each group. Mice in AST‐L group and AST‐H group were administered intragastrically with AST at 30 and 90 mg/kg/day, respectively, starting at 16–20 months. The mice in adult group and ageing group were given with 1% sodium carboxyl methylcellulose as the vehicle.

### 2.2 Measurement of oxygen consumption and carbon dioxide production

The oxygen (O_2_) consumption and carbon dioxide (CO_2_) production rates in mice were measured with Oxylet apparatus. Before collection of data, mice were acclimatized in the measurement system for 1 week. After AST administration, O_2_ consumption and CO_2_ production rates of mice in four groups were monitored for nine consecutive weeks before the mice were sacrificed. The volume of O_2_ consumption (VO_2_) and the volume of CO_2_ release (VCO_2_) were recorded every 5 min. The respiratory quotient (RQ) = VCO_2_/VO_2_ was then calculated.

### 2.3 Isolation and culture of primary hepatocytes of mice

Isolation and culture of primary hepatocytes of mice were performed according to the method previously reported in the literature.^27^ Briefly, after mice were anaesthetized, 50 ml of perfusion buffer (Krebs Ringer buffer containing 3.6 mg/ml glucose, 1 M calcium chloride and 0.66 mg/ml collagenase I) was used. Hepatocytes were isolated through the enzymatic perfusion with collagenase of portal vein at 37°C. The mouse liver was transferred to a 10‐cm cell culture dish containing 20 ml of cold collagenase‐free perfusion solution under aseptic conditions. The isolated liver was sliced, and the hepatocytes were dispersed by pipetting with large holes and filtered with 70‐μm cell strainer into a 50‐ml centrifuge tube and centrifuged at 50 *g* at 4°C for 2 min. The supernatant was removed, and then, the pellet cells were washed twice with 50% Percoll; Cold HepatoZYME‐SFM (Gibco; 15 ml) was used to suspended the pellet, which was supplemented with 2 mM l‐glutamine, 20 units/ml penicillin and 20  μg/ml streptomycin. After cell viability was checked with placental blue staining, hepatocytes (1 × 10^6^ cells/well) were seeded into a 6‐cm cell culture dish pre‐covered with collagen and then cultured in M199 medium containing 10% foetal bovine serum (FBS) for subsequent experiments.

### 2.4 Measurement of the levels of serum insulin and leptin and levels of serum and hepatic triglyceride

The serum insulin and leptin levels were measured with the Mouse Adiponectin Magnetic Bead kit according to manufacturer's instructions. The measurement was performed with the Plex MAGPIX reader of Bio‐Rad laboratories, and TG levels in serum and hepatic homogenate were assayed with TG Determination Kit (BioVision) according to the instructions.

### 2.5 Assays of mRNA levels of the related genes with quantitative real‐time PCR

Total RNA was extracted from mouse liver tissue or isolated hepatocytes with TRIzol reagent (Invitrogen) according to the instructions of the reagent. After being treated with DNase, RNA integrity was tested with 1.2% agarose gel electrophoresis. The RNA concentration was measured with UV spectrophotometer at a wavelength of 260 nm (OD_260_) and OD_280_. The purity of the isolated RNA samples was indicated by the ratio of OD_260_/OD_280_, which was equal to or higher than 1.8. Reverse transcription was performed with 2 μg of total RNA to synthesize cDNA template. The qRT‐PCR was performed as follows: 1 μl of cDNA sample solution (diluted 1:5), 1 μl of specific primers, 10 μl of SYBR Green PCR Master Mix and a final volume of 20 μl. The initial reaction was at 95ºC for 10 min, followed by 40 cycles at 95°C for 15 s and 60°C for 1 min. The relative expression level of gene was analysed by the 2^−ΔΔCt^ method, using GAPDH as an internal control. The PCR‐specific primers were listed in Table 1.

**TABLE 1:** The primer sequences used for real‐time PCR

Gene	Forward primer	Reverse primer
ACS	gcctgggtgggaaagtcc	gcagtgcactcggtctgt
CPT1a	gatcctggacaatacctcggag	ctccacagcatcaagagactgc
CPT1b	ggaggtggctttggtccc	ggcggatgtggttcccaa
CACT	gccaacgctgcctgtttc	cttcctcctcctgcccct
ECHS	aagcccagttcggacagc	gcggtcaccagtgaggac
ACADM	agctctagacgaagccacga	tgagcctagcgagttcaacc
HMGCS2	cccaagggctgtggactg	caggggagcaggagggat
cytochrome *b*	agtgcgtgttgctcgacaa	gcggtgtgcagtgctatcat
12S rRNA	ccaccgcggtcatacgatta	ttgggtcttagctgtcgtgt
18S	tagagggacaagtggcgttc	cgctgagccagtcagtgt
GAPDH	aactttggcattgtggaagg	acacattgggggtaggaaca

### 2.6 Detection of the related proteins with Western blot

The liver tissue or isolated hepatocytes were homogenized with radioimmunoprecipitation assay (RIPA) buffer (RIPA lysate: phenylmethylsulfonyl fluoride: protein phosphatase inhibitor = 100:1:1). The homogenate was centrifuged at 12,000 *g*, 4°C for 15 min. The supernatant was taken and saved. After protein concentration was measured with bicinchoninic acid solution (BCA) methods, protein sample solutions (50 μg/lane) were diluted with 5 × loading buffer and heated at 100°C for 5 min and then electrophoresed in 10% sodium dodecyl sulphate‐polyacrylamide gel electrophoresis (SDS‐PAGE) gel. The gel was then transferred to polyvinylidene fluoride (PVDF) membrane, blocked with 5% milk for 1 h, 4°C and then incubated with the corresponding primary antibody overnight at 4°C. The membrane was washed three times with 1 × Tris‐buffered saline, 0.1% Tween® 20 Detergent (TBST) buffer for three times, and then incubated with the corresponding secondary antibody at room temperature for 1 h. The targeted protein band of membrane was developed by incubating with ECL chemiluminescent solution. Image‐Pro Plus 6.0 software was used to analyse the intensity of band images. The following corresponding antibodies were used in this study: hormone‐sensitive lipase (HSL) antibody (Abcam, ab45422, 1: 1000), phosphorylated HSL antibody (Abcam, ab109400, 1: 500), adipose TG lipase (ATGL) antibody (Abcam, ab207799, 1: 1000), acetyl‐CoA carboxylase (ACC1) antibody (Abcam, ab45174, 1:1000), phosphorylated ACC1 antibody (Abcam, ab68191, 1: 1000), AMP‐activated protein kinase (AMPK) antibody (Abcam, ab110036, 1:2000), phosphorylated AMPK antibody (Abcam, ab129081, 1: 1000), carnitine palmitoyltransferase 1a (CPT1a) antibody (Abcam, ab234111, 1: 1000), carnitine palmitoyltransferase 1b (CPT1b) antibody (Abcam, ab87773, 1: 1000), carnitine‐acylcarnitine translocase (CACT) antibody (Abcam, ab224388, 1: 1000), ACS antibody (Abcam, ab177958, 1: 1000), enoyl coenzyme A hydratase‐short chain (ECHS) antibody (Abcam, ab170108, 1: 1000), acyl‐coenzyme A dehydrogenase (ACADM) antibody (Abcam, ab92461, 1:1000) and 3‐hydroxy‐3‐methylglutaryl coenzyme A synthase‐2 (HMGCS2; Abcam, ab137043, 1: 1000).

### 2.7 Lipolysis test and malonyl‐CoA assay

Fifteen micrograms of isolated mouse visceral fat tissue was put into 100 μl of lipolysis buffer (Krebs buffer with 0.1% glucose and 3.5% fatty acid‐free BSA) in a 96‐well plate and incubated at 37°C with shaking at 450 rpm for 2 h. The amount of glycerol released in the culture medium was assayed with Lipolysis Colorimetric Assay Kit (Millipore Sigma) according to the instructions of the manufacturer. The content of malonyl‐CoA in liver tissue was detected with malonyl‐CoA ELISA kit (MyBioSource). Tissue homogenization, processing testing and result analysis were all carried out according to the instructions.

### 2.8 Fatty acid β‐oxidation test

The isolated hepatocytes were seeded into a 24‐well extracellular flux (XF) culture plate. After incubation for 3 h, the medium was replaced with XF alkaline medium containing 5.5 mM glucose and 50 μM carnitine. 150 μM deuterium‐labelled palmitate was used to stimulate the maximum oxygen consumption rate (OCR) response.

### 2.9 Detection of oxygen consumption rate

Oxygen consumption rate was measured at 37°C with XF96 extracellular analyser (Seahorse Bioscience). The procedures were briefly described as follows: after the isolated hepatocytes were seeded and incubated for 3 h, they were washed with XF alkaline medium, and the tested medium was pre‐equilibrated at 37°C without CO_2_ for 1 h. When 0.5 μM oligomycin and 1 μM carbonyl cyanide‐p‐trifluoromethoxyphenylhydrazone (FCCP) were sequentially added, 1 μM rotenone and antimycin A were finally added, and the OCR was measured under alkaline conditions.

### 2.10 Detection of plasma β‐hydroxybutyrate and assay of ATP content

The content of plasma β‐hydroxybutyrate was detected with the LiquiColor end detection kit according to the instructions. Briefly, 6 μl of standard or plasma samples was added to 251 μl of R1 working solution (heated at 37°C), and the baseline level was immediately read spectrophotometrically at a wavelength of 505 nm, followed by adding 38 μl of R2 reagent and incubation at 37°C for 5 min. The amount of end product was measured by reading at 505 nm (OD_505_) again. The plasma β‐hydroxybutyrate content was calculated based on the standard curve. ATP levels in isolated hepatocytes or liver tissues were measured with ATP kit (Promega) according to the instructions. The data were normalized to protein levels.

### 2.11 Isolation of mitochondria

After the mouse liver was quickly removed, the liver mitochondria were isolated by differential centrifugation. Briefly, the liver was manually homogenized with a glass homogenizer and centrifuged at 400 *g* at 4°C for 10 min, and the supernatant was saved and centrifuged at 9000 *g* at 4°C for 10 min. The mitochondrial pellet was suspended with storage buffer. The mitochondrial protein concentration was determined with BCA methods as described above.

### 2.12 Detection of the activities of mitochondria respiratory chain complexes

The isolated hepatocytes were lysed with lysis buffer (250 mM sucrose, 5 mM Tris‐HCL, 2 mM ethylene glycol‐bis(β‐aminoethyl ether)‐N,N,N′,N′‐tetraacetic acid [EGTA]) at 4°C. The lysate was centrifuged at 4°C at 760 *g* for 10 min. The supernatant was saved and re‐centrifuged at 8740 *g* for 10 min at 4°C. The pellet was suspended with lysis buffer and centrifuged again at 8460 *g* for 10 min at 4°C. Rotenone‐sensitive NADH‐ubiquinone reductase was used as a substrate to detect complex I activity. Malonate‐sensitive succinate‐ubiquinone reductase was used as a substrate to detect the activity of complex II. Antimycin‐sensitive ubiquinone‐cytochrome *C* reductase was used as a substrate to detect the activity of complex III. Cytochrome *C* cyanide‐sensitive cytochrome *C* oxidase was used as a substrate to detect the activity of complex IV. All the assays were performed in triplicate at 37°C.

### 2.13 Detection of mitochondrial DNA content

In order to quantify mitochondrial DNA (mtDNA) content of primary hepatocytes, we used NucleoSpin kit (Macherey‐Nagel) to extract total genomic DNA and then used real‐time PCR to detect two mtDNA‐specific sequences, namely cytochrome *b* (MT‐CYB) and 12S rRNA, using 18S as a nuclear DNA control. The primer sequences for PCR were listed in Table 1.

### 2.14 Statistical analysis

All the data are expressed as mean ± standard deviation (SD). The experimental data were analysed and processed with statistic software, including SPSS13.0 and Image‐Pro Plus 6.0. The significance of the difference between the means of each group was determined by single‐factor variance analysis (one‐way ANOVA) to test, *p* < 0.05 indicates that the difference is statistically significant.

## 3 RESULTS

### 3.1 The effects of AST on metabolic parameters of ageing mice

To examine the effects of AST on lipid metabolism of ageing mice, we measured several lipid metabolism‐related parameters. We firstly examined its effects on body weight (Figure 1A), visceral fat (Figure 1B) and liver weight (Figure 1C), and then calculated the ratio of visceral fat and liver to body weight. We also measured the levels of serum TG (Figure 1D), hepatic TG (Figure 1E) and serum insulin (Figure 1F). The results showed that as compared with those of the adult group, the body weight, the visceral fat and the ratio of liver to body weight of the ageing mice were all increased significantly (*p* < 0.05; Figure 1A–C). As compared with those of the ageing group, after being treated with AST, the body weight, visceral fat and liver‐to‐body weight ratio of the mice were significantly reduced dose‐dependently (*p* < 0.05; Figure 1A–C). As compared with those of mice in the adult group, the levels of serum TG and hepatic TG of the ageing mice were increased significantly (*p* < 0.05; Figure 1D,E). As compared with those of the ageing group, the levels in the serum TG and hepatic TG of the mice after being treated with AST were significantly reduced in a dose‐dependent manner (*p* < 0.05; Figure 1D,E). Additionally, as compared with those of mice in the adult group, the levels of serum insulin of the mice in ageing group were also significantly increased (*p* < 0.05; Figure 1F,G). As compared with those of mice in ageing group, the levels of serum insulin after being treated with AST were significantly reduced in a dose‐dependent manner (*p* < 0.05; Figure 1F,G). After H&E staining, in the ageing liver, there was much lipid droplet; however, they were decreased after AST treatment. In the ageing adipose tissue, the size of adipocytes was larger than that of adult group, which decreased when AST treatment. In line with these results observed by H&E staining, Oil red staining displayed that there was much lipid accumulation in the ageing liver and adipose tissue, which decreased after AST treatment dose‐dependently (Figure S1).

**FIGURE 1:** The effects of Astragaloside IV (AST) on the metabolic parameters of ageing mice. The body weight (A), visceral fat (B), liver weight (C) and body weight ratio of mice in each group were measured. The contents of triglyceride (TG) in serum (D) and liver (E) of mice were also measured. Fasting serum insulin level (F) was indicated. Data are expressed as mean ± SD. *p < 0.05, **p < 0.01 (*n *= 10)

### 3.2 The effects of AST administration on lipolysis, lipase and respiratory quotient in ageing mice

Since the results shown in Figure 1 indicated that AST treatment can significantly reduce the levels of serum TG and hepatic TG, in order to determine whether AST has an effect on lipolysis (the hydrolysis of TGs into glycerol and fatty acids), we next detected the release of its backbone glycerol from ex‐vivo adipose tissue using the methods described previously.^28^ We measured the glycerol release. The results shown in Figure 2A indicated that as compared with that of mice in the adult group, the glycerol release from the visceral adipose tissue of the mice in ageing group after fasting was significantly reduced. As compared with that of the ageing group, the glycerol release from the visceral adipose tissue of AST‐treated mice was significantly increased after fasting with that in mice of AST‐H group being higher than that in AST‐L group (*p* < 0.05; Figure 2A). Lipolysis is mainly catalysed by ATGL and HSL. Next, we examined the effect of AST on the protein expression levels of HSL, phosphorylated HSL (pHSL) and ATGL in the visceral adipose tissue of adult and ageing mice with Western blot. The results indicated that as compared with those of the mice in adult group, the protein levels of pHSL and ATGL in visceral adipose tissue of ageing mice were significantly reduced. As compared with those of mice in ageing group, after AST administration, the protein levels of ATGL and pHSL in visceral adipose tissue of ageing mice were significantly increased in a dose‐dependent manner (*p* < 0.05; Figure 2B) but the protein level of HSL was not significantly changed among these groups (Figure 2B). In order to reflect the effect of AST administration on energy expenditure, we monitored the changes in mouse RQ, that is the volume ratio of mouse CO_2_ to O_2_ (CO_2_/O_2_), which can be used to estimate the type of fuel utilization.^29^ The obtained results showed that as compared with those of the mice in adult group, RQ of mice in ageing group was significantly higher. After being treated with AST, RQ of ageing mice was significantly decreased in a dose‐dependent manner (*p* < 0.05; Figure 2C)

**FIGURE 2:** The effects of Astragaloside IV (AST) on lipolysis, lipase and respiratory quotient (RQ) in ageing mice. (A) The release of glycerol from visceral adipose tissue of mice in each group. (B) The phosphorylation status and the total protein levels of HSL and ATGL of visceral adipose tissue of mice in each group detected by Western blot. (C) The average weekly change in respiratory quotient (RQ) at 9 weeks after AST administration. The results are expressed as mean ± SD, *p < 0.05, ^#^ *p* < 0.05 vs ageing group (*n* = 10)

### 3.3 AST induced the shift of hepatic lipid catabolism in ageing mice

AMP‐activated protein kinase (AMPK) is a metabolic regulator, which can enhance insulin sensitivity and FAO. In order to explore the potential mechanism for reducing RQ, an indicator of the shift of lipid utilization by the organisms, we examined the levels of AMPKα, phosphorylated AMPKα (pAMPKα) as well as its downstream target ACC1 and phosphorylated ACC1 (pACC1) in mouse liver. We also measured the content of the product of ACC1, malonyl‐CoA (Malonyl‐CoA). We observed that in the liver of ageing mice, while the expression levels of AMPK in adult and ageing mice were not significantly different, the level of pAMPK was significantly lower in ageing mice than that of adult mice. After being administrated with AST, its phosphorylation was significantly increased, and the ratio of pAMPK to total AMPK was also significantly increased in a dose‐dependent manner (*p* < 0.05; Figure 3A), indicating the phosphorylated activation of AMPK by AST.

**FIGURE 3:** Astragaloside IV (AST) increased the levels of phosphorylated AMPK and ACC1 in the liver of ageing mice and reduced the content of malonyl‐CoA. (A) Representative Western blot results of AMPK, ACC1, phosphorylated AMPK and ACC1. The histogram shows the ratio of phosphorylated AMPK to AMPK, and the ratio of phosphorylated ACC1 to ACC1. (B) The reduced malonyl‐CoA levels caused by AST treatment. The results are expressed as mean ± SD, and statistical significance is indicated as *p < 0.05, **p < 0.01, ***p < 0.001 (*n *= 10)

AMPK is the upstream inhibitor of ACC1, which catalyses the carboxylation of acetyl‐CoA to generate malonyl‐CoA, a key step in fatty acid biosynthesis. Thus, we examined the effects of AST on the expression levels of ACC1 and phosphorylated ACC1(pACC1). We found that in the liver of ageing mice, while the expression levels of ACC1 were not significantly different between adult mice and ageing mice, the expression level of pACC1 was significantly lower in ageing mice than that in adult mice. After being administrated with AST, the level of pACC1 was significantly increased, and the ratio of phosphorylated ACC1 to total ACC1 was also significantly increased dose‐dependently (*p* < 0.05; Figure 3A), indicating that ACC1 is inhibited. Consistent with these findings, we observed that the level of ACC1 product, malonyl‐CoA, was significantly higher in ageing mice than that in adult mice, and AST treatment could also significantly reduce the level of malonyl‐CoA in the liver of ageing mice (*p* < 0.05; Figure 3B), partially explaining the above‐mentioned switch from fatty acid biosynthesis to fatty acid oxidation.

### 3.4 AST promoted fatty acid activation and mitochondrial transport in the liver of ageing mice

Fatty acids must be activated prior to being oxidized; that is, acyl‐CoA synthetase (ACS) catalyses the formation of acyl‐CoA. The activated acyl‐CoA must enter the mitochondria where it is further oxidized. Long‐chain acyl‐CoA cannot directly penetrate mitochondrial inner membrane. It needs to be synthesized with carnitine under the catalysis of CPT1a to form acyl carnitine, which then enters the mitochondrial matrix through the inner membrane under the catalysis of CACT. The fatty acyl carnitine that enters the mitochondria is converted into fatty acyl‐CoA under the action of CPT1b in the inner mitochondrial membrane. In order to determine the effects of AST on hepatic fatty acid activation and mitochondrial transport in ageing mice, we tested whether AST could affect the expression levels of ACS, CPT1a, CPT1b and CACT at both the mRNA level with qRT‐PCR and protein levels with Western blot. We found that the mRNA levels (Figure 4A) and protein levels (Figure 4B) of ACS, CPT1a, CPT1b and CACT were all significantly lower in mice in ageing group than in adult group. Administration of ageing mice with AST significantly and dose‐dependently up‐regulated the expression levels of ACS, CPT1a, CPT1b and CACT in the liver of ageing mice at both mRNA level (Figure 4A) and protein level (Figure 4B; *p* < 0.05).

**FIGURE 4:** Astragaloside IV (AST) increased the expression levels of the enzymes involved in fatty acid activation and transport in the liver of ageing mice. (A) The effect of AST on the mRNA expression levels of ACS, CPT1a, CPT1b and CACT in the liver of ageing mice. (B) The effect of AST on the protein expression levels of ACS, CPT1a, CPT1b and CACT in the liver of ageing mice. The results are expressed as mean ± SD, and statistical significance is indicated as *p < 0.05, **p < 0.01, ***p < 0.001 (*n *= 10)

### 3.5 AST promoted fatty acid β‐oxidation and ketone body production in hepatocytes of ageing mice

To further explore the effects of AST on lipid catabolism, we examined the effects of AST on oxidation of deuterium‐labelled palmitate in primary hepatocytes isolated from ageing mice and AST‐treated mice. We observed that when primary hepatocytes were incubated with deuterium‐labelled palmitic acid‐BSA conjugate, the deuterium was released from palmitic acid and integrated into water. In this way, the oxidation rate of palmitic acid could be calculated from the production of deuterium‐labelled water in the medium. We monitored the palmitic acid release rates of mice in adult, ageing, ageing + AST‐L and ageing + AST‐H groups at 24 and 48 h. At 24 h, the palmitic acid release rate of mice was significantly lower in ageing group than in adult group. After being administrated with AST, palmitic acid release rate of ageing mice was significantly increased dose‐dependently as compared to that of ageing mice without being administrated, and similar effect was also observed at 48 h (Figure 5A). Etomoxir is an irreversible inhibitor of carnitine acyltransferase 1, which can inhibit the entry of fatty acids into mitochondria, thereby inhibiting β‐oxidation of fatty acids. In our experiment, we observed that after co‐incubating primary hepatocytes with AST and 100 μM Etomoxir, the palmitic acid oxidation of primary hepatocytes from ageing mice and AST‐treated ageing mice was significantly reduced, and the effect of AST on enhancing palmitic acid oxidation disappeared (Figure 5B), indicating that AST enhances palmitic acid oxidation through mitochondrial FAO.

**FIGURE 5:** Astragaloside IV (AST) promoted fatty acid β‐oxidation and ketone body production in hepatocytes of ageing mice. (A) After AST treatment, the hepatocytes of mice in each group were isolated and cultured for 24 and 48 h. The oxidation of deuterium‐labelled palmitate was detected. (B) After ageing mice were administrated with AST, the primary hepatocytes isolated from liver of mice in each group were incubated with 100 μM etomoxir for 48 h, and the oxidation of deuterium‐labelled palmitate was detected. (C) The effects of AST on the mRNA expression levels of ECHS and ACADM in hepatocytes of mice in each group. (D) The effects of AST on the protein expression levels of ECHS and ACADM in hepatocytes of mice in each group. (E) The effect of AST on the level of plasma β‐hydroxybutyrate in ageing mice under basic conditions and fasting for 24 h. (F) The effects of AST on the mRNA and protein expression levels of HMGCS2 in the liver of mice when fasting for 24 h. The results are expressed as mean ± SD, and statistical significance is indicated as *p < 0.05, **p < 0.01, ***p < 0.001 (*n *= 10)

To further confirm the effect of AST on FAO, we tested the effects of AST on the enzymes involved in FAO in hepatocytes, including the changes in expression levels of ECHS and ACADM. We found that the mRNA levels (Figure 5C) and protein levels (Figure 5D) of ECHS and ACADM were lower in mice in ageing group than in adult group and that administration of ageing mice with AST significantly up‐regulated the expression levels of ECHS and ACADM in hepatocytes of ageing mice at both mRNA (Figure 5C) and protein levels (Figure 5D), respectively, (*p* < 0.05), confirming that AST can promote FAO in hepatocytes of ageing mice.

A large amount of acetyl‐CoA produced by FAO in the liver can be partially converted into ketone bodies, including about 30% acetoacetate, about 70% β‐hydroxybutyrate and trace amounts of acetone. To further test whether AST can exert its effect on the production of ketone bodies in the liver, we measured the levels of serum β‐hydroxybutyric acid in ageing mice and AST‐treated ageing mice. We found that under basal conditions, there was no difference in serum β‐hydroxybutyric acid levels in mice among all four groups (Figure 5E), but after fasting for 24 h, as compared with that of mice in the adult group, the serum β‐hydroxybutyric acid levels of ageing mice were significantly decreased. After being treated with AST, the serum β‐hydroxybutyric acid level of ageing mice was significantly increased dose‐dependently (Figure 5E; *p* < 0.05). To explore how AST regulates the production of ketone bodies, we focused on examining the effects of AST on the expression levels of HMGCS2, the rate‐limiting step of KB production. We found that the hepatic expression level of HMGCS2 was significantly lower in ageing mice than in adult mice (Figure 5F). However, after being treated with AST, the mRNA and protein expression levels of HMGCS2 in the liver of ageing mice were significantly increased in a dose‐dependent manner (Figure 5F; *p* < 0.05).

### 3.6 AST enhanced the mitochondrial functions of hepatocytes in ageing mice and enhanced their biosynthesis capacities

In order to evaluate the effect of AST on the mitochondrial functions of hepatocytes in ageing mice, we measured the basal and maximum mitochondrial respiration rate, which represents the OCR. As compared with those of the adult group, the basal and maximum mitochondrial respiration rates of hepatocytes in ageing mice were decreased significantly, and administration of ageing mice with AST resulted in a significant increase in the basal and maximum mitochondrial respiration rates (Figure 6A; *p* < 0.05).

**FIGURE 6:** Astragaloside IV (AST) enhanced the mitochondrial functions and promoted mitochondrial biosynthesis capacity of hepatocytes in ageing mice. (A) Oligomycin (0.5 μM), carbonyl cyanide‐p‐trifluoromethoxyphenylhydrazone (FCCP) (1 μM), rotenone (1 μM) and antimycin A (1 μM) at the indicated time points were sequentially added to hepatocytes isolated from mice in each group, and the mitochondrial function was reflected by measuring the basial and maximum oxygen consumption rates (OCRs) of the cells. (B) Relative ATP levels and ADP/ATP ratios in the isolated hepatocytes and liver tissues of mice in each group. (C) The activities of mitochondrial electron transport chain complexes I, II, III and IV of hepatocytes were normalized to mitochondrial protein (mg). (D) Copy numbers of MT‐CYB and 12S rRNA genes. The results are expressed as mean ± SD, and statistical significance is indicated as *p < 0.05, **p < 0.01 (*n *= 10)

In order to further explore whether the stimulating effects of AST on mitochondrial respiration rates are related to the regulation of cellular energy metabolism, we examined the effects of AST on ATP level and the ratio of ATP/ADP in hepatocytes isolated from mice with bioluminescence analysis. As compared with that of the mice in adult group, the ATP level in the hepatocytes of ageing mice was decreased by approximately 35%. However, the reduction in ATP level was significantly attenuated in ageing mice after being administrated with AST. Further experiments in mice also found that compared with the adult mice, the ATP content in the liver tissue of ageing mice was also significantly reduced, and after being administrated with AST at high‐dose, this attenuation could be significantly improved (Figure 6B; *p* < 0.05). To further confirm the effects of AST on mitochondrial respiratory chain (MRC) functions, we examined the activities of the MRC of the isolated hepatocyte. As shown in Figure 6C, as compared with those of the adult group, the activities of complexes I, II, III and IV in the liver of ageing mice were significantly reduced. After being administrated with AST, this reduction in MRC activities could be effectively and significantly reversed in a dose‐dependent manner (Figure 6C; *p* < 0.05). MT‐CYB and 12S rRNA are two mtDNA‐encoded genes, and their copy numbers are closely related to mitochondrial biosynthesis.^30^ Thus, we examined the effects of AST on copy numbers of mtDNA‐encoded MT‐CYB and 12S rRNA genes. Our results indicated that as compared with those of adult group, the copy numbers of MT‐CYB and 12S rRNA genes in the hepatocytes of ageing mice were significantly reduced, but were significantly increased in a dose‐dependent manner after being administrated with AST. Consistent with this, AST administration could also significantly promote mitochondrial biosynthesis capacity as the results of increasing mtDNA replications, which was reflected by the increasing copy numbers of mtDNA‐encoded MT‐CYB and 12S rRNA genes (Figure 6D; *p* < 0.05). In conclusion, these results indicate that AST can regulate lipid metabolisms and energy metabolism in healthy ageing mice by regulating mitochondrial functions and biosynthesis capacity of liver cells.

## 4 DISCUSSION

The ageing population is increasing worldwide. The mechanisms underlying ageing process involve many genetic, biochemical, physiological, nutritional and environmental factors and their interactions. During the ageing process, abnormal lipid metabolism and energy metabolism are one of the important alterations of many biochemical and physiological parameters.^31^ In the present study, we examined the effects of AST on biochemical and physiological parameters related to lipid metabolism pathways and the enzymes/proteins involved in these pathways, including fatty acid biosynthesis and fatty acid β‐oxidation, KB production, mitochondrial electron transport chain (ETC) and mitochondrial biosynthesis capacity in hepatocytes and liver of ageing mice. Our results indicate that AST administration stimulated FAO and KB production by up‐regulation of the key enzymes/proteins involved in these two processes and inhibited fatty acid biosynthesis by down‐regulating the enzymes/proteins involved in this pathway. The key findings were discussed as follows.

We first examined the effects of AST on the biochemical and physiological parameters, including body weight, visceral fat, liver weight, the ratio of visceral fat and liver to body weight, levels of serum TG and hepatic TG, serum insulin, which are related to lipid metabolism pathways in hepatocytes and liver of ageing. We found that they were all significantly enhanced by AST administration (Figure 1). These results indicate that AST can reverse the alterations of ageing‐induced metabolic parameters in mice. It has been shown that in the process of ageing, the effect on lipolysis of visceral adipose tissue is weakened.^32^ Lipolysis refers to the process in which TGs are hydrolysed into FFAs and glycerol under the action of lipase and cofactors, including perilipin‐1 (PLIN1). Among them, ATGL and HSL are the most important lipases involved in the lipolysis process, and they control about 95% of lipolysis of lipids. The results of the current study showed that AST administration could significantly enhance the release of glycerol from fat tissue of ageing mice after fasting, indicating that AST administration can enhance the lipolysis of adipose tissue of ageing mice. Our further experimental results show that the enhancing effects of AST on lipolysis are mainly related to its effects on up‐regulation of the expression levels of ATGL and the phosphorylated form of HSL (pHSL; Figure 2). RQ refers to the ratio of CO_2_ volume to O_2_ volume in mice, which can be used as an indicator to evaluate the body's utilization of raw materials. Our results showed that after AST administration, the average RQ of ageing mice was significantly reduced (Figure 2), indicating that AST administration can significantly promote the body's utilization of lipids and regulate energy metabolism. The liver is an important site for regulating lipid metabolism. The characteristic manifestation of the disorders of lipid metabolism in the body caused by ageing is the accumulation of TGs in the liver. AST administration can significantly reduce the ratio of liver weight to body weight and reduce hepatic TG content (Figure 1), indicating that the liver plays an important role in AST‐mediated regulation of lipid metabolism. AMPK is an important regulator of hepatic lipid metabolism, which can enhance insulin sensitivity and fatty acid oxidation.^33^ Our results showed that AST administration could significantly enhance the expression of pAMPK in the liver of ageing mice (Figure 3), indicating that AST can activate AMPK in the liver. ACC1 is the downstream target of AMPK and can catalyse the production of malonyl‐CoA. After AST administration, the level of the phosphorylated ACC1 (pACC1) in the liver of ageing mice was enhanced, and a decrease in malonyl‐CoA content was also detected (Figure 3), indicating that AST treatment results in phosphorylation of ACC1 by activating liver AMPK to reduce its activity.

In this study, we found AST promoted ATP generation. Thus, we confirmed that AST could enhance energy metabolism. AMP‐activated protein kinase (AMPK) was a metabolic regulator, which involved mitochondrial biogenesis in response to energy deprivation. Generally, AMPK was activated when the cellular AMP/ATP ratio changed.

We found that AST administration increased mRNA and protein levels of several key enzymes/proteins, including ACS, CPT1a, CPT1b and CACT, involved in the activation of fatty acid and transport in the liver of ageing mice. After AST enhances the lipolysis of TGs of ageing adipose tissue, the fatty acids released from TGs must be activated; that is, acyl‐CoA synthetase (ACS) catalyses the production of acyl‐CoA before entering the mitochondria and being oxidized. When long‐chain fatty acyl‐CoA enters the mitochondria, it needs to be catalysed by CPT1a to generate fatty acylcarnitine, which is catalysed by CACT, enters the mitochondrial matrix through the inner membrane and then is converted into fatty acyl‐CoA under the action of CPT1b. Our results show that AST can up‐regulate the mRNA and protein levels of ACS, CPT1a, CPT1b and CACT in the liver of ageing mice (Figure 4), indicating that AST can promote the activation of fatty acids in liver cells of ageing mice and their transport into mitochondria.

We found that AST administration promoted mitochondrial FAO. Mitochondrial FAO is the main pathway to provide energy source for the body.^34^ The fatty acyl‐CoA that has entered the mitochondria is catalysed by the enzymes involved in FAO system, starting from the fatty acyl β‐carbon atom, and then undergoing a four‐step reaction of dehydrogenation, water addition, dehydrogenation and thiolysis to generate one molecule of acetyl‐CoA, that is fatty acyl‐CoA with fewer than two carbon atoms. These reactions are repeated to finally complete the β‐oxidation of fatty acids. In order to further explore the effect of AST on lipid catabolism during ageing, we first detected the effect of AST on palmitic acid oxidation in primary hepatocytes of ageing mice. We found that AST could enhance the FAO in hepatocytes of ageing mice (Figure 5). When the primary hepatocytes were co‐incubated with etomoxir, an inhibitor of carnitine acyltransferase 1, which inhibits the entry of fatty acids into mitochondria, the effect of AST on enhancing FAO disappeared (Figure 5), indicating that regulation of AST on FAO is closely related to mitochondria. Next, we examined the changes in expression levels of enzymes involved in FAO in hepatocytes, including ECHS and fatty ACADM. We found that AST could up‐regulate the mRNA and protein levels of both ECHS and ACADM in hepatocytes of ageing mice, respectively, (Figure 5), indicating that AST can enhance mitochondrial FAO in hepatocytes of ageing mice.

We found that AST administration promoted KB production. Acetyl‐CoA is one of the main products of FAO, and a part of acetyl‐CoA derived from FAO can be converted into ketone bodies in the liver. Our experiment found that AST could enhance serum level of β‐hydroxybutyric acid (one of the main components of ketone bodies) of ageing mice after fasting for 24 h. We also found that AST could up‐regulate both mRNA and protein levels of HMGCS2, the rate‐limiting enzyme that produces ketone bodies (Figure 5). These results further confirm that AST can enhance FAO and the subsequent KB production in liver of ageing mice.

We found that AST administration enhanced the mitochondrial ETC functions and promoted mitochondrial biosynthesis capacity of isolated hepatocytes and/or liver of ageing mice. Mitochondria play a key role in FAO and energy production. It has been reported that mitochondrial dysfunction in hepatocytes contributes to the occurrence of fatty liver disease. Therefore, maintaining normal mitochondrial function is very important for body health.^35^ In the current study, OCR was used to reflect MRC function. We found that AST administration could significantly increase the basal and maximum OCR of ageing mice, and increased ATP level in primary hepatocytes and liver tissues and enhanced the activities of ETC complexes I, II, III and IV (Figure 6). On the other hand, the copy numbers of mtDNA can also be used as a parameter for evaluating mitochondrial functions.^36^ Our results showed that AST administration could increase the copy numbers of two mtDNA‐encoded genes, MT‐CYB and 12S rRNA (Figure 6), indicating that AST can increase the mitochondrial ETC biogenesis and functions of hepatocytes.

Astragaloside IV has been known to possess a wide variety of medical and health beneficial effects, including anti‐viral, anti‐inflammation, antioxidant, anti‐hyperglycaemic, anti‐chromic asthma, gastroprotection, neuroprotection and anti‐apoptotic properties.^37^ The results obtained in this study clearly indicate that AST can have a beneficial effect on improving the abnormal lipid metabolism associated with ageing and that its action mechanisms mainly involve AMPK/ACC1/mitochondrial β‐oxidation signal axis as highlighted in Figure 7. Given the increasing prevalence of senile obesity associated with ageing, the current study has indicated that AST can be potentially used to prepare AST‐containing functional foods for the treatment of the abnormal lipid metabolism symptoms, and for alleviation of senile obesity associated with ageing for the elderly population. To the best of our knowledge, this is the first study investigating the effects of AST on healthy and natural ageing mice. Further studies to address its potential applications in the treatment of abnormal lipid metabolism symptoms and senile obesity are warranted.

**FIGURE 7:** Proposed model for the acting mechanisms underlying the regulation of mitochondrial energy metabolism of mice by Astragaloside IV (AST). AST exerts its role on metabolic regulation in healthy ageing mice, mainly by activating AMPK, which leads to the inhibition of ACC1 and activation of fatty acid β‐oxidation in mouse liver

Insulin is critical in fatty acid metabolism and a study reported that insulin reduces expression of ATGL and HSL through the GDF3‐ALK7 signalling pathway, resulting in inhibition of lipolysis.^38^ Insulin regulates the synthesis and storage of liver lipids partly by increasing lipogenesis by PI3K/PDK1 pathway and suppressing fatty acid oxidation.^39^ A study found that insulin increases the level of malonyl‐CoA to inhibit β‐oxidation of fat acids.^40^ Therefore, insulin can inhibit lipolysis and beta oxidation and promote synthesis. We found that AST treatment decreased the serum insulin, thus promoting lipolysis and beta oxidation, and inhibiting lipid synthesis.

## 5 CONCLUSIONS

In the current study, we have observed that AST enhances lipid catabolism in ageing mice by regulating the mRNA and protein expression levels of genes related to lipid metabolism and mitochondrial FAO in mouse liver. Our results also indicate that AST plays an important role in regulating the activities of MRC and energy metabolism as well as mitochondrial functions in ageing mice. Therefore, mitochondrial FAO can serve as a promising therapeutic target for using AST to treat the abnormal lipid metabolism during ageing.

## CONFLICT OF INTEREST

The authors declare that there are no conflicts of interest.

## AUTHOR CONTRIBUTIONS

**Zhixiao Luo:** Investigation (lead). **Yaqi Wang:** Investigation (supporting); Software (supporting). **Mengzhen Xue:** Investigation (supporting); Software (lead). **Fangqi Xia:** Investigation (supporting). **Leiqi Zhu:** Investigation (supporting). **Yuanyang Li:** Investigation (supporting); Software (supporting). **Dengke Jia:** Investigation (supporting); Software (supporting). **Silong Chen:** Data curation (supporting). **Guangfu Xu:** Data curation (supporting). **Yan Lei:** Conceptualization (lead); Writing‐review & editing (lead).

## Supporting information

Fig S1

## Data Availability

The data that support the findings of this study are available from the corresponding author upon reasonable request.
